# Nucleostemin expression in invasive breast cancer

**DOI:** 10.1186/1471-2407-14-215

**Published:** 2014-03-21

**Authors:** Takayuki Kobayashi, Kenkichi Masutomi, Kenji Tamura, Tomoyuki Moriya, Tamio Yamasaki, Yasuhiro Fujiwara, Shunji Takahashi, Junji Yamamoto, Hitoshi Tsuda

**Affiliations:** 1 Department of Basic Pathology, National Defense Medical College, 3-2 Namiki, Tokorozawa, Saitama 359-8513, Japan; 2 Department of Medical Oncology, Cancer Institute Hospital, 3-8-31 Ariake, Koto-ku, Tokyo 135-8550, Japan; 3 Division of Cancer Stem Cell, National Cancer Center Research Institute, Tsukiji, Chuo-ku, Tokyo 104-0045, Japan; 4 Department of Breast Oncology and Medical Oncology, National Cancer Center Hospital, 5-1-1 Tsukiji, Chuo-ku, Tokyo 104-0045, Japan; 5 Department of Surgery, National Defense Medical College, 3-2 Namiki, Tokorozawa, Saitama 359-8513, Japan; 6 Department of Pathology and Clinical Laboratories, National Cancer Center Hospital, 5-1-1 Tsukiji, Chuo-ku, Tokyo 104-0045, Japan

## Abstract

**Background:**

Recently, the cancer stem cell hypothesis has become widely accepted. Cancer stem cells are thought to possess the ability to undergo self-renewal and differentiation, similar to normal stem cells. Nucleostemin (NS), initially cloned from rat neural stem cells, binds to various proteins, including p53, in the nucleus and is thought to be a key molecule for stemness. NS is expressed in various types of cancers; therefore, its role in cancer pathogenesis is thought to be important. This study was conducted to clarify the clinicopathological and prognostic impact of NS in invasive breast cancers.

**Method:**

The correlation between NS immunoreactivity and clinicopathological parameters was examined in 220 consecutive surgically resected invasive breast cancer tissue samples by using tissue microarrays. The presence of nuclear NS and p53 immunoreactivity in 10% or more of cancer cells was considered as a positive result.

**Results:**

Among the 220 patients, 154 were hormone-receptor (HR)-positive, 22 HER2-positive/HR-negative, and 44 HR-negative/HER2-negative. One hundred and forty-two tumors (64.5%) showed NS positivity, and this positivity was significantly correlated with estrogen receptor (ER) (*P* = 0.050), human epidermal growth factor receptor 2 (HER2) (*P* = 0.021), and p53 (*P* = 0.031) positivity. The patients with NS-positive tumors showed significantly shorter disease-free survival than those with NS-negative tumors. Furthermore, the patient group with NS- and p53-positive tumors showed significantly poorer prognosis than other patient groups. Multivariate analysis showed that NS status was an independent prognostic indicator.

**Conclusions:**

NS may play a significant role in the determination of breast cancer progression in association with p53 alterations. The NS status of patients with luminal and HER2 type breast cancers may be a useful prognostic marker.

## Background

Breast cancer is one of the most prevalent diseases worldwide. While most patients with early breast cancers are cured with surgically resection followed by appropriate adjuvant drug and radiation therapy, approximately 30% of these patients experience relapse and develop metastatic disease [1]. In this metastatic stage, tumor cells frequently acquire resistance to various drugs during intensive systemic therapies, and eventually their aggressiveness and growth become uncontrollable. Less than 5% of patients with distant metastatic tumors live for 5 years [2]. Therefore, identification of potential targets with the aim of developing interventional drugs is an important area of research.

The hypothesis that various types of cancers, including breast cancer, are generated by a limited number of cancer stem cells has been widely accepted recently [3]. Cancer stem cells, like normal stem cells, are thought to have two important characteristics: the ability to undergo self-renewal and the ability to undergo differentiation into different cell types [4]. Furthermore, these cells are thought to be inherently resistant to various therapeutic drugs, making the eradication of tumors containing cancer stem cells with the use of the current treatment protocols difficult [5]. To overcome these obstacles, the development of new therapeutic strategies to target cancer stem cells is essential for the management of breast cancer.

Nucleostemin (NS) is thought to be a key molecule for maintaining “stemness” [6]. NS was initially cloned from rat neural stem cells and was found to contain two GTP-binding motifs and an N-terminal basic domain, which is essential for binding to p53 [6]. NS accumulates mainly in the nucleoli and moves to the nucleoplasm after binding with GTP. Interaction of NS with a multitude of proteins in the nucleoplasm, including p53, may play a significant role in self-renewal, cell cycle regulation, apoptosis, and cell proliferation [7].

NS is expressed in central nervous system stem cells, embryonic stem cells, and primitive cells in the bone marrow and testes [6]. Furthermore, various types of cancers, including the following, have been reported to express NS: squamous cell carcinomas of the uterine cervix; head, neck, esophagus, and renal cell carcinomas; and prostate cancer [8-13]. Moreover, recent evidence indicates that NS is involved in maintaining cancer stem cells [14,15]. These findings suggest that NS may also play an important role in cancer pathogenesis as well as in cancer stem cell maintenance. However, no clinical study has investigated the role of NS in breast cancer.

If NS is expressed in breast cancer stem cells and its expression is correlated with disease progression in breast cancer, it may serve as a powerful prognostic marker for clinical use. To test this hypothesis, we investigated the expression of NS in surgically resected invasive breast cancer specimens from 220 patients by using immunohistochemistry. Furthermore, we examined the prognostic implication of the combination status of NS and p53 and the significance of NS expression status among the three biological subtypes of breast tumors: (a) hormone-receptor (HR) positive (luminal type); (b) human epidermal growth factor receptor 2 (HER2) positive (HER2 type); and (c) HR negative and HER2 negative (triple negative).

## Methods

### Patients and tumor specimens

The patient cohort used in the present study was the same as the cohort reported in our previous study [16]. Briefly, formalin-fixed paraffin-embedded tissue blocks of invasive breast cancer specimens from 220 consecutive patients were used to construct tissue microarrays (TMAs). All patients with unilateral invasive breast carcinoma underwent mastectomy or breast-conserving surgery at the National Defense Medical College (NDMC) Hospital, Tokorozawa, Japan from 1995 through 1999. These patients had a median follow-up of 74 months after surgery (range, 1–151 months), during which 58 patients experienced relapse. Of the 220 patients, 218 were female patients and 2 were male patients; 101 (45.9%) patients had lymph node metastasis and 8 (3.6%) had distant metastasis at the time of breast cancer diagnosis. In most cases, patients with hormone receptor-positive tumors at the time of diagnosis were prescribed adjuvant endocrine therapy (e.g., tamoxifen, toremifene, fadrozole, or LHRH analogues) for two or more years. The patients with a large tumor and/or four or more lymph node metastases received one of the following adjuvant chemotherapy regimens: cyclophosphamide-epirubicin-5-fluorouracil (CEF), cyclophosphamide-adriamycin-5-fluorouracil (CAF), cyclophosphamide-methotrexate-5-fluorouracil (CMF), and oral fluoropyrimidines. Detailed patient and disease characteristics are documented in Table 1. Clinicopathological data were retrospectively obtained from medical records [16].

**Table 1:** Correlation between nucleostemin expression and clinicopathological variables in surgically resected breast cancers

**Variable**		**Number of cases (%)**		
		**Nucleostemin expression**		
	**Total**	**Positive**	**Negative**	**P-value**
	**(n = 220)**	**(n = 142)**	**(n = 78)**	
Age				
Median (range)		52 (30 ~ 82 y)		
≦52	109	71 (65)	38	0.89
>52	111	71 (64)	40	
Tumor size				
<5.0 cm	174	108 (62)	66	0.21
≧5.0 cm	42	31 (74)	11	
Unknown	4	4(100)	0	
Lymph node metastasis				
Negative	115	70 (61)	45	0.39
Positive	101	68 (67)	33	
Unknown	4	4 (100)	0	
Distant metastasis				
Negative	209	134 (64)	75	0.72
Positive	8	6 (75)	2	
Unknown	3	2 (67)	1	
Stage				
I or II	179	111 (61)	68	0.13
III or IV	37	28 (76)	9	
Unknown	4	3 (75)	1	
Nuclear grade				
1, 2	137	86 (63)	51	0.48
3	83	56 (67)	27	
ER status				
Negative	88	50 (57)	38	0.050
Positive	132	92 (70)	40	
PgR status				
Negative	96	57 (59)	39	0.16
Positive	124	85 (69)	39	
HR (ER/PgR) status				
Negative	66	40 (61)	26	0.42
Positive	154	102 (66)	52	
HER2 status				
Negative	190	117 (62)	73	0.02
Positive	30	25 (83)	5	
p53 status				
Negative	143	85 (59)	58	0.03
Positive	77	57 (74)	20	
Histological type				
Ductal	191	125 (65)	66	0.38
Lobular	10	5 (50)	5	
Mucinous	6	6 (100)	0	
Tubular	5	1 (20)	4	
Medullary	3	2 (67)	1	
Other	5	3 (60)	2	

*Abbreviation:ER* Estrogen receptor, *PgR* Progesterone receptor, *HR* Hormone receptor.

This study was approved by the Medical Ethical Committee of National Defense Medical College and by the Institutional Review Board of National Cancer Center.

### Tissue microarray construction

We constructed TMA blocks as previously described [16]. Briefly, double tissue cores with a diameter of 2 mm were obtained from each donor block, and these core specimens were transferred to a recipient block using a Tissue Microarrayer (Beecher Instruments, Silver Spring, MD, USA). One TMA block contained a maximum of 26 tumor samples, and 13 TMA sets were used in this study.

### Immunohistochemistry

Immunohistochemistry was performed on TMA sections of 220 patients. The antibodies used were mouse monoclonal anti-human NS (clone BL2858; Bethyl Laboratories, Inc., Montgomery, TX, USA) and mouse monoclonal anti-human p53 (clone DO-7; Dako, Carpinteria, CA, USA). Formalin-fixed paraffin-embedded specimens on the TMA were cut into 4 μm-thick sections. The tissue sections were deparaffinized twice in xylene for 10 min and rehydrated through graded ethanol (99%, 90%, 80%, and 70%) to water. Antigens were retrieved by microwave heating for 30 min in 10 mM sodium citrate (pH 6.0) for NS and by autoclaving for 15 min in 10 mM Tris–HCl (pH 9.0) for p53. To block endogenous peroxidase activity, the sections were treated with 100% methanol containing 3% hydrogen peroxide for 5 min. Non-specific binding was blocked by incubation in 2% normal swine serum (Dako) in phosphate-buffered saline. The slides were incubated with primary antibodies at 4°C overnight and then reacted with a dextran polymer reagent combined with secondary antibodies and peroxidase (Envision Plus; Dako) for 30 min at room temperature. Specific antigen–antibody reactions were visualized with 0.2% diaminobenzidine tetrahydrochloride and hydrogen peroxide. Counterstaining was performed using Mayer’s hematoxylin. A separate assay was run using a case of esophageal carcinoma as a positive control for NS [17]. Reactions without the primary antibodies were used as negative controls.

NS and p53 expression was assessed according to the proportion of nuclear staining area. Specimens with 10% or more immunoreactive tumor cells were considered positive, and those with less than 10% were considered negative. Immunohistochemistry results were independently evaluated by two observers (T.K. and H.T.), and cases with discrepant grades were re-evaluated by discussion until consensus was achieved.

ER, PgR, and HER2 had already been immunohistochemically re-assessed on new sections in our previous study [16] by using mouse monoclonal anti-human ER (clone 1D5, Dako), mouse anti-human PgR (clone PgR636, DAKO), and rabbit polyclonal anti-HER2 antibody (HercepTest kit, Dako) according to the methods recommended by the manufacturer. ER and PgR were considered positive if the nuclear staining was observed in 10% or more of tumor cells. Samples were considered hormone receptor positive if they were ER and/or PgR positive and hormone receptor negative if they were ER and PgR negative. HER2 results were considered positive if the IHC score was “3+” or gene amplification was detected by FISH according to the 2007 ASCO/CAP guideline [18].

### Statistical analysis

Comparisons between groups were evaluated using chi-squared test or Fisher’s exact test. Disease-free survival (DFS) curves of patients were drawn using the Kaplan-Meier method and compared using the log-rank test. Cox multivariate proportional hazards models were used to explore the association of variables with DFS. For all tests, *P* < 0.05 was considered to be statistically significant. All analyses were performed using the software JMP 6.0 for Windows (SAS Institute Inc., Cary, NC, USA).

## Results

### Clinicopathological and prognostic implications of NS expression for the entire patient cohort

Initially, the expression levels of NS were classified as negative (0%), weak (1% to <10%), moderate (10% to <30%), or strong (30% or more). The number of cases categorized into the negative, weak, moderate, and strong groups was 62, 16, 55, and 87, respectively. From these results, we judged that NS expression showed bimodal distribution and used a 10% threshold for NS positivity between negative and positive groups.

NS protein was frequently detected in the nucleus of breast cancer cells. Although strong immunoreaction was observed in both the nucleoli and nucleoplasm of cancer cells (Figure 1A), nuclear immunoreaction of NS in some cases was limited to the nucleoli of cancer cells (Figure 1B). Such cells were also judged as positive for NS immunoreactivity. Cytoplasmic staining was not observed. These findings are consistent with those of previous reports [6,17,19]. We found that 78 (35.5%) or 142 (64.5%) patients had NS-negative or NS-positive tumors, respectively (Figure 1C). Unremarkable mammary glands showed nuclear NS immunoreactivity in almost all luminal epithelial cells (Figure 1D).

**Figure 1:** **Nucleostemin (NS) expression in human breast cancer tissues. A**. A NS-positive tumor. Almost all cancer cells show NS immunoreactivity in both nucleoli and nucleoplasm. **B**. Another NS-positive tumor, NS immunoreactivity is limited to nucleoli in nuclei of cancer cells. Such cancer cells are also judged as NS-positive. This case was also classified as NS-positive. **C**. A NS-negative tumor. **D**. An unremarkable mammary gland shows nuclear NS immunoreactivity in almost all luminal epithelial cells.

Tumors with NS positivity showed a higher frequency of ER positivity, HER2 positivity, and p53 positivity (*P* = 0.050, *P* = 0.021, and *P* = 0.031, respectively), whereas NS expression status was not correlated with tumor size, lymph node metastasis, distant metastasis, tumor nuclear grade, or PgR positivity. NS expression was detected at 50% or more in all histological types studied except tubular carcinoma (20%), and the positive rate was 100% (6 of 6) in mucinous carcinoma. Patients with NS-positive tumors showed significantly shorter DFS time than those with NS-negative tumors (*P* = 0.020, Figure 2).

**Figure 2:** **Prognostic impact of NS status in the patients with primary breast cancer.** This figure shows disease-free survival (DFS) curves for the 142 patients with NS-positive tumors and for the 78 patients with NS-negative tumors. These two curves differ significantly (*P* = 0.020).

### Prognostic implication of the NS and p53 combination status for the entire patient cohort

Since it has been reported that physical and functional interaction between NS and p53 appear to be essential for self-renewal, cell cycle regulation, cell proliferation, and apoptosis [7], we next examined the prognostic implication of the combination status of NS and p53 for the entire patient cohort. We found that 143 (65%) and 77 (35%) patients had p53-negative and p53-positive tumors, respectively. The patients with p53-positive tumors showed significantly shorter DFS time than those with p53-negative tumors (*P* = 0.006, Figure 3A).

**Figure 3:** **Prognostic impact of the combination status of NS and p53 in the patients with primary breast cancer. A**. Disease-free survival (DFS) curves for the 77 patients with p53-positive tumors and for the 143 patients with p53-negative tumors. These two curves differ significantly (*P* = 0.006). **B**. This figure shows three disease-free survival (DFS) curves: for the 57 patients with NS-positive and p53-positive tumors (‘unfavorable group’), for 105 patients comprising 20 NS-negative and p53-positive tumors and 85 NS-positive and p53-negative tumors (‘intermediate’ group), and for 58 patients with NS-negative and p53-negative tumors (‘favorable’ group). The unfavorable group has significantly shorter DFS time than the intermediate group or the favorable group (log-rank test *P* = 0.034 and *P* = 0.0007, respectively).

A striking stratification of relapse risk was identified when three different combinations of NS and p53 status were evaluated: 57 cases with a combination of NS-positive/p53-positive tumors (unfavorable group); 105 cases comprising 20 NS-negative/p53-positive tumors and 85 NS-positive/p53-negative tumors (intermediate group); and 58 cases with NS-negative/p53-negative tumors (favorable group). The unfavorable group had a 5-year DFS rate of 55%, compared with 75% in the intermediate group and 86% in the favorable group (Figure 3B). The unfavorable group had significantly shorter DFS time than the intermediate and favorable groups (log-rank test *P* = 0.034 and *P* = 0.0007, respectively).

### Prognostic implication of NS among the three biological subtypes of breast tumors

Currently, treatment strategies differ between the biological subtypes of breast tumors; therefore, we examined the prognostic implication of NS among three groups of patients divided based on their biological subtype: 154 patients with luminal-type tumors (HR-positive); 22 patients with HER2-type tumors (HER2-positive and HR-negative); and 44 patients with triple-negative tumors (HR and HER2-negative). Eight patients with HR-positive and HER2-positive tumors were included and analyzed as luminal-type patients.

Among the patients with luminal-type tumors, patients with NS-positive tumors showed a significantly shorter DFS time than those with NS-negative tumors (*P* = 0.033, Figure 4A). Among the patients with HER2-positive tumors, patients with NS-positive tumors had a 5-year DFS rate of 28% compared with 100% in patients with NS-negative tumors (Figure 4B). However, the *P*-value was not calculated because there was no relapse in the four patients with NS-negative tumors. Among the patients with triple-negative tumors, there was no difference between the survival curves for patients with NS-positive tumors and those with NS-negative tumors (*P* = 0.41, Figure 4C).

**Figure 4:** **Prognostic impact of NS status in the three subgroups of the different biological subtype tumors: luminal-type tumors, HER2-type tumors, and triple-negative tumors. A**. Subgroup analysis of the 154 patients with luminal-type tumors (HR-positive tumors). Two disease-free survival (DFS) curves, that for the 102 patients with NS-positive tumors and that for the 52 patients with NS negative tumors, differ significantly (*P* = 0.033). **B**. Subgroup analysis of the 22 patients with HER2-type tumors (HER2-positive and HR-negative tumors). In two disease-free survival (DFS) curves, that for the 18 patients with NS-positive tumors and that for the 4 patients with NS-negative tumors, five-year DFS rates differ largely (100% vs 28%). *P*-value was not available because there was no relapse in the patients with NS-negative tumors. **C**. Subgroup analysis of the 44 patients with triple-negative tumors (HR and HER2 negative tumors). The two curves do not differ significantly (*P* = 0.41).

### Multivariate analysis of prognostic factors and evaluation of NS

Univariate analysis showed that HR, HER2, nuclear grade, tumor size, nodal status, distant metastasis, and NS expression were significantly correlated with DFS. When multivariate analysis was performed using these seven factors, NS expression status was selected as an independent prognostic factor (*P* = 0.036), together with nuclear grade, tumor size, lymph node status, and distant metastatic status (*P* = 0.0008, 0.0007, 0.0038 and <0.0001, respectively; Table 2).

**Table 2:** Prognostic impacts of clinicopathological variables computed by Cox’s univariate and multivariate analyses in patients with primary breast cancer

		**Univariate**			**Multivariate**		
		**Hazard ratio**	**(95% CI)**	**P-value**	**Hazard ratio**	**(95%CI)**	**P-value**
**Disease free survival**							
Nucleostemin	Negative	1		0.023	1		0.036
	Positive	2.06	(1.11-3.84)		2.13	(1.05-4.33)	
Hormone-receptor	Positive	1		0.045	1		0.46
	Negative	1.73	(1.01-2.95)		0.78	(0.39-1.52)	
HER2	Negative	1		0.0005	1		0.17
	Positive	2.91	(1.59-5.34)		1.65	(0.80-3.41)	
Nuclear grade	1, 2	1		<0.0001	1		0.0008
	3	3.30	(1.94-5.64)		2.97	(1.57-5.61)	
Tumor size	≦5.0 cm	1		<0.0001	1		0.0007
	>5.0 cm	6.89	(3.97-11.9)		2.99	(1.59-5.66)	
Nodal status	Negative	1		<0.0001	1		0.0038
	Positive	4.51	(2.45-8.31)		2.73	(1.38-5.38)	
Distant metastasis	Negative	1		<0.0001	1		<0.0001
	Positive	71.6	(26.1-196.5)		62.3	(15.5-251.1)	

*Abbreviation:* 95% CI 95% confidence interval.

## Discussion

In the present cohort, we found that the NS protein expression status was positively correlated with both ER and HER2 status and was a powerful prognostic factor. Patients with NS-positive breast tumors had a significantly shorter DFS time than those with NS-negative tumors (*P* = 0.020, Figure 2), and multivariate analysis for DFS showed that NS positivity had an independent impact as a prognostic indicator among breast cancer patients (*P* = 0.036, Table 2). To our knowledge, this is the first report to show the clinical implication of NS protein expression in invasive breast cancers.

Although several studies have shown the important roles of NS in the pathogenesis of various cancer types [8-13] as well as the maintenance of cancer stem cells [14,15], no direct evidence is yet available to support that NS is a marker of cancer stem cells. Currently, molecules such as CD44, CD133, ALDH1, and CXCR4 have been found to be potential markers of cancer stem cells [20-25]. Furthermore, the expression of these stem cell markers has been shown to be a poor prognostic indicator in several human cancer types [24,26-30]. Based on these observations, our results show that high NS expression is a powerful indicator of poor outcome, consistent with the idea that NS may be a breast cancer stem cell marker.

The limitations of the present study included the retrospective analyses and the heterogeneity of adjuvant treatments. Therefore, one should pay careful attention when interpreting these results. Further studies using a uniformly treated patient cohort are required to clarify the role of NS in breast cancer stem cells.

We found that the patient group with tumors coexpressing NS and p53 had shorter DFS times than the patient group with tumors negative for either NS or p53. GTP binding modulates the movement of NS from the nucleoli to the nucleoplasm; NS then binds p53 at its N-terminal basic domain, which results in the suppression of p53 function [6,7]. Because prolongation of the half-life of most of the mutated p53 protein induces its nuclear accumulation, it is generally believed that the p53 pathway does not fully function in tumors with high p53 nuclear immunoreactivity [31-33]. This evidence leads to the assumption that p53 function would be profoundly suppressed in tumors coexpressing NS and p53. Our results show the validity of this concept and that functional crosstalk between NS and p53 may also occur *in vivo*.

Currently, we cannot explain the correlation between NS expression and p53 expression. Although several studies have shown that NS modulates the expression of wild-type p53 [34,35], the role of NS in breast cancers with mutant p53 has not yet been evaluated. Further research is needed to elucidate the correlation.

We found that the NS expression status was positively correlated with both ER and HER2 status and also found a significant prognostic implication of NS expression for patients with luminal-type tumors and those with HER2-type tumors, except for those with triple-negative tumors. NS was first identified as a gene upregulated in MCF-7 cells upon 17β-estradiol treatment [36]; therefore, our inclusion of subgroup analysis among patients with luminal-type tumors was reasonable. To our knowledge, this is the first report to demonstrate the possible association between NS and HER2. Zhang G et al. showed that NS is required for the expression of EGF and EGFR in an esophageal squamous carcinoma cell line [13]. Presumably, NS is required for the expression of HER2 in a manner similar to that for EGFR. We found no survival impact of the NS expression status among patients with triple-negative tumors, who show higher rates of mutated p53 than patients with luminal-type or HER2-type tumors [37]. NS can function in the presence of wide-type p53 [7]; therefore, the expression status of NS may have survival impact only for the luminal-type and HER2-type tumors.

## Conclusions

In summary, our results indicate that the expression status of NS, abundant in stem cells, is a prognostic indicator in breast cancer patients, especially for those with luminal-type or HER2-type tumors, and that the coexpression of NS and p53 correlates with poorer prognostic outcomes. Examination of NS expression may be useful for the stratification and management of breast cancer patients in future daily practice.

## Competing interests

The authors declare no conflicts of interest.

## Authors’ contributions

TK and HT conceived of the study, performed experiments, analyzed data and wrote the manuscript. TM, TY, and JY provided samples, collected clinical and pathological data. KM, KT, YF, and ST participated in designing the study and revising the manuscript. HT participated in the overall design and study coordination and finalized the draft of the manuscript. All authors read and approved the final manuscript.

## Pre-publication history

The pre-publication history for this paper can be accessed here:

http://www.biomedcentral.com/1471-2407/14/215/prepub
